RETRACTED

# Effects of Insulin Combined with Traditional Chinese Medicine Assisted Comprehensive Nursing Intervention on Oxidative Stress State, Cell Adhesion Factor, and Pregnancy Outcome of Patients with Gestational Diabetes Mellitus

**DOI:** 10.1155/2022/5330134

**Published:** 2022-04-06

**Authors:** Yanling Zhou, Bei Yang, Rongrong Yao, Ping Sun

**Affiliations:** ^1^Department of Obstetrics, Yantaishan Hospittal, Yantai 264000, China; ^2^Outpatient Department, Qingdao Eighth People's Hospital, Qingdao 266100, China; ^3^Traditional Chinese Medicine Department, The Affiliated Qingdao Central Hospital of Qingdao University, The Second Affiliated Hospital of Medical College of Qingdao University, Qingdao 266042, China; ^4^Department of Obstetrics, The Affiliated Qingdao Central Hospital of Qingdao University, The Second Affiliated Hospital of Medical College of Qingdao University, Qingdao 266042, China

## Abstract

**Objectives:**

The changes of oxidative stress state, cell adhesion factor (sICAM-1) level, blood glucose, and blood lipid of patients with gestational diabetes mellitus (GDM) assisted by insulin combined with traditional Chinese medicine (TCM) prescription were detected to explore the effect of TCM treatment on maternal and infant outcomes of GDM.

**Methods:**

A total of 60 patients diagnosed with GDM from January 2019 to December 2019 were selected. Among them, 30 patients were treated with insulin combined with TCM prescription (control group), and 30 patients were treated with nursing intervention based on control group (study group). Serum of maternal vein and fetal umbilical vein was collected. The contents of superoxide dismutase (SOD) and lipid oxide (MDA) were determined. The content of intercellular adhesion factor (ICAM-1) was measured, and the differences of fasting blood glucose (FPG), glycosylated hemoglobin (HbA1c), triglyceride (TG), cholesterol (CHO) and low density lipoprotein (LDL-C) between 2 groups were compared. The incidence of maternal and infant adverse outcomes was assessed.

**Results:**

After treatment, blood glucose indexes in 2 groups were decreased, and the study group was lower than the control group. After treatment, LDL-C, TC and TG in 2 groups were lower than before, and the study group was lower than the control group. HDL-C was higher than before treatment, and the study group was higher than the control group. After treatment, oxidation-related substances SOD and GSH-Px in 2 groups were higher than before, and those in study group were higher than those in control group. ROS and MDA were lower than before treatment, and the level of sICAM-1 in the study group was significantly higher than that in the control group. Clinical application of insulin combined with TCM prescription assisted comprehensive nursing intervention in the treatment of gestational diabetes, pregnancy outcome is improved.

RETRACTED

**Conclusions:**

Oxidative stress imbalance exists in GDM and the causes of adverse pregnancy outcomes are closely related to oxidative stress and vascular endothelial injury. TCM can improve the oxidative stress imbalance and the pregnancy outcome of patients with GDM from the perspective of reducing vascular endothelial injury. Comprehensive nursing intervention for pregnant women with GDM can optimize the outcome of pregnancy and is worthy of clinical application.

## 1. Introduction

GDM refers to diabetes or abnormal glucose tolerance that occurs or is first detected during pregnancy [1, 2]. With changes lifestyle, food structure and metabolites during pregnancy, the incidence of GDM increased year by year [3, 4]. The incidence of GDM is reported to be 1%∼14% in various countries, and it is reported that the incidence of GDM in China is about 1%∼ 5% [5]. GDM has a great influence on mothers and children. The recent effects are mainly urinary and reproductive infections, polyhydramnios, hypertension during pregnancy, and ketoacidosis in pregnant women, peripheral blood oxidation and antioxidant dysfunction, fetal impact can lead to fetal malformation, abortion, stillbirth, fetal giant, fetal growth restriction, and neonates are prone to hypoglycemia and respiratory distress syndrome [6–10]. The long-term effects are as high as 30%∼60% of patients with gestational diabetes relapse during the second pregnancy [11], 50% within 7 years, and 75% within 24 years to develop type 2 diabetes or impaired glucose tolerance [12–14]. Moreover, the risks of offspring physical development, intelligence and neurobehavioral development, metabolic abnormalities and chronic diseases are affected to a certain extent.

Due to the particularity of GDM patients, it is difficult to treat them. The goal of treatment is to stabilize her blood sugar to a manageable level that meets the energy requirements of pregnancy while avoiding hypoglycemia and ketoacidosis. With the continuous development of perinatal medicine in recent years, the treatment options for gestational diabetes patients have gradually diversified. As one of them, insulin can accelerate the glycolysis and oxidation of glucose, promote glycogen synthesis, storage and fat conversion, thereby reducing maternal blood sugar, and the drug does not pass through the placenta, it has a good preventive effect on adverse neonatal outcomes to a certain extent [15, 16]. However, the effect of blood pressure control in some patients is not satisfactory [17].

RETRACTED

According to TCM, GDM belongs to the category of “pregnancy quench thirst,” and the treatment should focus on strengthening the spleen, raising the clear, nourishing the Yin and supplementing qi, paying attention to the spleen and stomach, coordinating the rise and fall of qi, so as to achieve the purpose of regulating subtle metabolism [18]. Simultaneous Chinese herbal formula combined with insulin therapy, Chinese medicine can stimulate B cells to secrete insulin, increase the body's use of sugar, and increase the number or affinity of insulin receptors, increase insulin sensitivity, and reduce insulin resistance effect. At the same time, patients with gestational diabetes are prone to stress, fear, anxiety and other negative emotions, which may lead to elevated blood glucose and aggravate the disease. Therefore, it is necessary to carry out targeted comprehensive nursing intervention for patients with this disease. Usually, for the psychological counseling of patients, it is necessary to conduct a comprehensive and comprehensive analysis of their current psychological state, provide a reasonable diet, choose a reasonable exercise method [19], improve bad living habits [20], provide a quiet and comfortable hospital environment, and provide family support therapy, so that get more systematic support to relieve or eliminate tension and anxiety symptoms [21, 22].

In this study, insulin combined with TCM prescription assisted comprehensive nursing intervention was used to explore the effects of insulin combined with TCM prescription assisted comprehensive nursing intervention on oxidative stress state, cell adhesion factor and pregnancy outcome of gestational diabetes mellitus from the perspective of oxidative stress.

## 2. Materials and Methods

### 2.1. The Research Object

Sixty patients with GDM admitted to our hospital from January 2019 to December 2019 were selected as the subjects of this study. Patients who had obtained informed consent were included in this study after the approval of the ethics Committee of our hospital.

#### 2.1.1. Inclusion Criteria

(1) Confirmed by blood glucose monitoring and urine glucose test, meeting the diagnostic criteria of gestational diabetes in 8th edition of Obstetrics and Gynecology; (2) no metabolic diseases such as diabetes before pregnancy; (3) the program was approved by the ethics Committee of the hospital, and patients voluntarily participate in it and sign informed consent.

#### 2.1.2. Exclusion Criteria

(1) Complicated with heart and lung dysfunction; (2) BMI >27 kg/m^2^; (3) complicated with pregnancy hypertension and other serious complications; (4) associated with pregnancy diseases such as placenta previa and threatened abortion; (5) poor treatment compliance; (6) adverse pregnancy history.

RETRACTED

### 2.2. Therapeutic Method

Dietary and exercise guidance and insulin subcutaneous injection therapy were given to patients in the two groups. Namely, calorie calculation was carried out based on standard weight and gestational age, and dietary control and exercise guidance were given to patients, who were told to eat more soy products, fruits and vegetables, eggs, milk, fish and lean meat, and eat less and more meals to effectively control blood glucose. 0.5 h after meals every day, exercise guidance such as walking and health exercises should be given to patients. During this period, patients' heart rate should be maintained at 120 times per minute, and exercise should be appropriate for 30 min a day. At the same time, insulin should be injected subcutaneously 15 ∼ 30 min before meals, and the dose should be gradually increased based on the patient's condition, blood glucose level and urine glucose level. For sensitive patients, the dose can be maintained at 5–10 U daily. Some obese and insensitive patients can adjust the dose according to the results of blood glucose test. At the same time, the patient was treated with self-made Chinese medicine prescription, which was composed of radix astragali seu hedysari (60 g), rehmannia glutinosa libosch (30 g), anemarrhenae rhizome (30 g), puerariae lobamle radix (30 g), ophiopogonis radix (20 g), polygonati odorati rhizome (20 g), lycii fructus (10 g), scutellariae radix (10 g) and phellodendri chinensis cortex (10 g), decocted and taken in water, 1 dose per day, 200 mL of juice, divided into 2 warm doses, if there are signs of delivery, stop taking.

On the basis of the control group, study group received comprehensive nursing intervention, including psychological nursing, diet intervention, exercise guidance, health education and medication guidance. Psychological nursing intervention is to actively communicate with pregnant women, to have a detailed understanding of the maternal history of pregnant women, to guide pregnant women to actively express their inner worries and concerns, to comfort and encourage pregnant women, and to explain all kinds of worries in pregnant women with clinical treatment. This can effectively improve their anxiety, tension and other negative emotions, actively and easily cope with the disease, and improve clinical compliance. At the same time, pregnant women who have already given birth are invited to speak out, to enhance their self-confidence in the disease, and pay attention to communicating with the pregnant woman's husband, asking the husband to comfort and understand the pregnant woman attentively, so that she can feel the warmth of the family and avoid bad emotions.

RETRACTED

## 3. Observation Target

### 3.1. Blood Glucose and Blood Lipids

Before and 4 weeks after treatment, fasting plasma glucose (FPG), 2 h postprandial blood glucose (2 h PBG), glycosylated hemoglobin (HbA1c), cholesterol (CHO), low density lipoprotein (LDL-C) and triglyceride (TG) levels in both groups were measured by PUZS-300 automatic biochemical analyzer.

FBG was measured by glucose oxidase. Glycated hemoglobin was determined by electrophoresis. Fasting insulin (FINS) was detected by solid phase competitive chemiluminescence ELISA. The levels of triglyceride (TG), cholesterol (CHO), high density lipoprotein cholesterol (HDL-C) and low density lipoprotein cholesterol (LDL-C) were determined by automatic biochemical analyzer.

### 3.2. Oxidative Stress State Detection

At two time points before and 2 weeks after treatment, 5 mL of fasting venous blood was collected from the patients, the centrifugal radius was set at 8 cm and the rotation speed was set at 3500 r/min, and the serum was collected. Malondialdehyde (MDA) was determined by thiobarbituric acid method (TBA). Determination of superoxide dismutase (SOD) was performed by xanthine oxidase method.

### 3.3. Cell Adhesion Factor

At two time points before and 2 weeks after treatment, 5 mL of fasting venous blood was collected from the patients, the centrifugal radius was set at 8 cm and the rotation speed was set at 3500 r/min, and the serum was collected. Soluble intercellular adhesion factor (sICAM-1) was determined by enzyme-linked reaction adsorption assay.

### 3.4. Pregnancy Outcomes

The maternal and infant outcomes of GDM pregnant women in the two groups were analyzed and compared, including cesarean section rate, postpartum related complications and newborn situation. Hyperhydramnios, premature rupture of membranes, cesarean section and abortion were observed in the two groups.

### 3.5. Statistical Analysis

The test index data of patients in the two groups were expressed as $\bar{x}\pm s$, and processed by SPSS 22.0 statistical analysis software. ANOVA or Chi-square test was used for comparison of differences between different groups, and *T* test was used for data test between the same groups. *P* < 0.05 was considered statistically significant.

## 4. Results

### 4.1. The General Information

The intrauterine gestation weeks at enrollment were 9 at 24 weeks, 12 at 25 weeks, 10 at 26 weeks, 14 at 27 weeks, and 15 at 28 weeks. The average intrauterine pregnancy was 26.15 weeks. Presences of labor were observed in all patients in this study. Patients were retrospectively divided into control group and study group. The control group consisted of 30 patients, aged from 21 to 38 years, with an average of 30.64 ± 4.30 years. In the study group, 30 patients were 22 to 40 years old, with an average of 31.53 ± 4.22 years old. There were no significant differences in age, body mass and gestational age among all patients, which were comparable (Table 1). The earlier the occurrence of hyperglycemia during pregnancy, the greater the impact on pregnant women and the fetus, the worse the prognosis, so it should be treated as soon as possible after diagnosis.

RETRACTED

### 4.2. Comparison of Blood Glucose Metabolism before and after Treatment

Before treatment, there were no significant differences in serum HbA1c (%), FPG (mmol/L), and 1 h PBG (mmol/L) and 2 h PBG (mmol/L) levels between 2 groups (Figure 1). Levels of serum HbA1c, FPG, 1 h PBG and 2 h PBG in 2 groups before delivery were significantly decreased versus those before treatment (Figure 1). Levels of serum HbA1c, FPG, 1H PBG and 2 h PBG in the study group were significantly lower than those of control group before delivery (Figure 1).

### 4.3. Comparison of Lipid Metabolism before and after Treatment

Before treatment, there was no significant difference in serum LDL-C, TC, TG, CHO, and HDL-C levels between the two groups (Figure 2). *T* test showed improvements in total cholesterol, triglyceride, and LDL cholesterol in both groups after treatment. After treatment, LDL-C, TC and TG in 2 groups were decreased, and observation group was lower than control group (Figure 2). HDL-C in 2 groups was higher than before treatment, and the study group was higher than the control group (Figure 2).

### 4.4. Comparison of Oxidative Stress State before and after Treatment

There were no significant differences in serum SOD, GSH-Px, ROS and MDA levels between the two groups before treatment (Figure 3). After treatment, SOD and GSH-Px in 2 groups were increased, and observation group was higher than control group (Figure 3). ROS and MDA in 2 groups were decreased, and the observation group was lower than the control group (Figure 3). The results showed that the level of oxidative stress determines the pregnancy outcome of gestational diabetes, and the increase of oxidative hyperproducts and the weakening of antioxidant defense ability are important reasons for the occurrence of complications in patients with advanced gestational diabetes, which may also be the pathophysiological mechanism of the occurrence of gestational diabetes and complications.

### 4.5. Comparison of Cell Adhesion Factor Content before and after Treatment

ICAM-1 belongs to the immunoglobulin superfamily with a molecular weight of 80000–14400. In diabetic patients, endothelial cells are activated due to HbA1c stimulation. Meanwhile, the immune stimulation of cytokines such as TNF and INF in blood stimulates endothelial cells to express ICAM-1, which is released into serum after endothelial cell necrosis. The level of sICAM-1 was significantly increased, and the level of sICAM-1 was proportional to the degree of vascular injury. The prognosis of gestational diabetes mellitus is related to the occurrence of vascular diseases [23]. The results of this study showed sICAM-1 content in the study group were lower than that in the control group (Figure 4).

RETRACTED

### 4.6. Comparison of Pregnancy Outcomes

Compared with the control group, the incidence of cesarean section, premature rupture of membranes and pregnancy hypertension in the study group were all lower (Table 2). The incidence of maternal and infant adverse outcomes in the study group was significantly higher than that in the control group (Table 2).

## 5. Discussion

Before pregnancy, glucose metabolism of pregnant women with GDM was normal or there was only latent hypoglycemia. Among all pregnant women with diabetes, about 80% were diagnosed with GDM and the rest were classified as diabetes combined with pregnancy. GDM is a high-risk pregnancy, which causes great damage to maternal and newborn health. Therefore, active and effective treatment must be taken to control the disease. With improvement of people's living standards and lifestyle changes, GDM incidence is increasing year by year. The pathogenesis of GDM is not very clear at present, and it is generally believed to be related to abnormal adipocytokine secretion and insulin resistance [24].

GDM generally adopts western medicine treatment, routine diet control, appropriate exercise. The control of blood glucose by insulin alone requires a long time to adjust the dose and finally reach the qualified dose required by the individual. However, the clinical effect of these methods is still not ideal, after treatment, pregnant women often have a high rate of adverse pregnancy. The combination of TCM and WM can improve the inflammatory response and the imbalance between oxidation and antioxidant in peripheral blood of GDM patients through better control of blood glucose, and further reduce maternal and infant adverse pregnancy outcomes incidence and reduce the dosage of insulin. In this study, astragalus membranaceus is the king medicine, sweet and mild, and belongs to the spleen and lung meridian, with the curative effect of supplementing the middle and benefiting qi. Astragalus can increase the synthesis of insulin signaling protein, promote the lowering of blood sugar, enhance the body's immunity and stress ability, and improve the heart function. Rehmannia glutinosa libosch contains rehmannia polysaccharide, which has the effect of beneficial qi, clearing heat, generating fluid, nourishing Yin and nourishing blood, affecting liver sugar metabolism, protecting vascular endothelium and reducing oxidative damage during the interaction between insulin and antagonistic hormones. Anemarrhenae rhizoma clearing heat and relieving fire, shengjin Runzao, can treat stomach heat quench thirst, bone steaming hot flashes. Puerariae lobamle radix can relieve fever, promote secretion of insulin B cells, and improve sensitivity of insulin receptor. Polygonati odorati rhizoma and phellodendri chinensis cortex can increase immunity, promote secretion of islet cells, and nourish qi, Yin and reduce blood sugar.

RETRACTED

In this study, insulin combined with TCM assisted comprehensive nursing intervention was used for the comprehensive treatment of gestational diabetes. The results showed that LDL-C, TC, TG, ROS and MDA levels in the study group after treatment were decreased versus control group. HDL-C, oxidation-related substances SOD, GSH-Px and sICAM-1 levels were increased versus control group. In the study group, insulin combined with TCM assisted comprehensive nursing intervention can significantly improve the blood glucose status and pregnancy outcome of patients with gestational diabetes. The reasons for this may be related to the effective control of blood glucose level and improvement of body immunity by insulin combined with TCM assisted comprehensive nursing intervention.

To sum up, simple drug therapy cannot achieve ideal results. Therefore, TCM therapy should be supplemented with comprehensive and standardized comprehensive nursing intervention in clinical treatment, such as guidance in diet, life and exercise, so as to better control the weight and blood sugar level of pregnant women and reduce the incidence of maternal and infant complications. TCM can improve the oxidative stress imbalance of patients with gestational diabetes and improve the pregnancy outcome of patients with gestational diabetes from the perspective of reducing vascular endothelial injury. Comprehensive nursing intervention for pregnant women with gestational diabetes can optimize the outcome of pregnancy and is worthy of clinical application.

## Figures and Tables

**Figure 1:** Comparison of glucose metabolism indexes between the two groups before and after treatment $\left(\bar{x}\pm s\right)$. Note: compared with before treatment ^*∗*^*P* < 0.05; compared with control group ^#^*P* < 0.05.

**Figure 2:** Changes in blood lipid of the two groups before and after treatment. Note: compared with before treatment ^*∗*^*P* < 0.05; compared with control group ^#^*P* < 0.05.

RETRACTED

**Figure 3:** Comparison of oxidation-related substances between the two groups before and after treatment. Note: compared with before treatment ^*∗*^*P* < 0.05; compared with control group ^#^*P* < 0.05.

**Figure 4:** Comparison of sICAM-1 content in maternal blood and umbilical cord blood between the two groups $\left(\bar{x}\pm s\right)$. Note: compared with control group ^#^*P* < 0.05.

**Table 1:** Comparison of general data between the two groups.

Group	Age	Body mass	Sampling of progesterone	Primipara/multipara
Control	30.64 ± 4.34	56.3 ± 5.5	11.9 ± 3.2	17/13
Study	31.53 ± 4.26	55.7 ± 5.6	11.3 ± 2.6	19/11
*t*/*χ*^2^	0.82	0.48	0.79	0.28
*P*	0.42	0.63	0.43	0.60

**Table 2:** Comparison of pregnancy outcomes between the two groups.

Group	Cesarean section	Amniotic fluid volume abnormality	Premature rupture of membranes	Pregnancy hypertension	Fetal distress	Threatened premature labor
Control	24 (80%)	4 (13.3%)	3 (10%)	4 (13.3%)	4 (13.3%)	3 (10%)
Study	5 (16.7%)	2 (6.7%)	2 (6.7%)	1 (3.3%)	1 (3.3%)	1 (3.3%)

## Data Availability

Data to support the findings of this study are available on reasonable request from the corresponding author.
